This article has been retracted.

# Design of Optimal Deep Learning-Based Pancreatic Tumor and Nontumor Classification Model Using Computed Tomography Scans

**DOI:** 10.1155/2022/2872461

**Published:** 2022-01-12

**Authors:** Maha M. Althobaiti, Ahmed Almulihi, Amal Adnan Ashour, Romany F. Mansour, Deepak Gupta

**Affiliations:** ^1^Department of Computer Science College of Computing and Information Technology, Taif University, P.O. Box 11099, Taif 21944, Saudi Arabia; ^2^Department of Oral & Maxillofacial Surgery and Diagnostic Sciences Faculty of Dentistry, Taif University, P.O. Box 11099, Taif 21944, Saudi Arabia; ^3^Department of Mathematics Faculty of Science, New Valley University, El-Kharga 72511, Egypt; ^4^Department of Computer Science & Engineering, Maharaja Agrasen Institute of Technology, Delhi, India

## Abstract

Pancreatic tumor is a lethal kind of tumor and its prediction is really poor in the current scenario. Automated pancreatic tumor classification using computer-aided diagnosis (CAD) model is necessary to track, predict, and classify the existence of pancreatic tumors. Artificial intelligence (AI) can offer extensive diagnostic expertise and accurate interventional image interpretation. With this motivation, this study designs an optimal deep learning based pancreatic tumor and nontumor classification (ODL-PTNTC) model using CT images. The goal of the ODL-PTNTC technique is to detect and classify the existence of pancreatic tumors and nontumor. The proposed ODL-PTNTC technique includes adaptive window filtering (AWF) technique to remove noise existing in it. In addition, sailfish optimizer based Kapur's Thresholding (SFO-KT) technique is employed for image segmentation process. Moreover, feature extraction using Capsule Network (CapsNet) is derived to generate a set of feature vectors. Furthermore, Political Optimizer (PO) with Cascade Forward Neural Network (CFNN) is employed for classification purposes. In order to validate the enhanced performance of the ODL-PTNTC technique, a series of simulations take place and the results are investigated under several aspects. A comprehensive comparative results analysis stated the promising performance of the ODL-PTNTC technique over the recent approaches.

## 1. Introduction

In recent years, pancreas tumor has been incurable and it is one of the deadliest diseases of which survival rates have not been greatly enhanced [1]. Currently, MRI guided radiation therapy is utilized for shrinking a tumor, but anatomical changes, like breathing, are unaffected due to the interpatient infarction and variability [2]. Accurate and earlier identification of the pancreatic tumor is a challenging task [3]. Enhancing early treatment, early diagnosis, and earlier detection is of greater significance. Computer-aided diagnosis (CAD) system was technologically advanced with the development of image processing and computer science technologies for detection and diagnosis. CAD system has been increasingly utilized by radiotherapists to improve diagnostic accuracy, assist in interpreting and detecting diseases, and reduce doctor pressure [4, 5].

CAD technique was newly created in a deep neural network (DNN) and extended the requirements for medical services. Higher pathology in pancreatic cancer leads to considerable attention in optimizing effective treatment and diagnostic CAD systems where correct pancreatic segmentation is needed [6]. Therefore, an innovative methodology of pancreatic segmentation needs to be developed. Now, computed tomography (CT) segmentation of the pancreas remains a challenge that is unresolved in the present study. The correct pancreatic segmentation in dice similarity coefficient (DSC) and CT scan on person without pancreatic lesion is increasingly complex due to the pancreatic segmentation with cancer lesion. Image recognition is the CAD's significant component. The procedure of recognizing adenocarcinomas consists of 2 stages: feature selection and feature extraction.

Image-guided treatment and image-based early diagnosis are the two emerging possible solutions. CT is widely employed for diagnoses and follow-ups in patients with PC. But, in up to 30%, a patient is wrongfully diagnosed with PC, or the diagnoses of PC are delayed. Image-guided treatment is capable of providing accurate targeting to improve curative options. Artificial intelligence (AI) could improve and provide accurate interventional image interpretation and extensive diagnostic expertise [7]. Current advancements have effectively been employed in imaging diagnosis tasks over radiology, dermatology, and ophthalmology. This advanced technology must be adaptable for the automated diagnosis of PC in CT scans. Possibly, AI technique is capable of providing a great deal of assistance in screening programs to identify the diseases in an early phase, thus increasing the efficiency of treatment.

Precise pancreatic segmentation is indispensable to generate annotated dataset for computer-assisted interventional guidance AI, as well as for development and training. The number of instances in the training dataset, that is, size of the dataset, also considerably influences the performance of the AI models [8]. Trained data needs precise outline of lesions and organs of interest. Any uncertainties in the outline would impact the performances in constrained dataset. In order to cover large numbers of pancreatic shapes and surrounding tissues, hundreds of thousands of CT scans should be annotated which are time-consuming. Interventional image guidance needs precise outline of the relevant anatomy and pancreas [9]. Automatic deep learning (DL) segmentation performances in CT pancreatic imaging are lower because of the complex anatomy and poor gray value contrast. The problem occurs because of an absence of contrast among pancreatic bowel and parenchyma, particularly with the duodenum. Furthermore, large variation in peripancreatic fat tissue and large variation in sizes of the pancreatic volume, over textural variation of the pancreatic parenchyma, also increase the complexity of the problem.

This study designs an optimal deep learning based pancreatic tumor and nontumor classification (ODL-PTNTC) model using CT images. The proposed ODL-PTNTC technique includes adaptive window filtering (AWF) technique to remove the noise existing in it. Besides, sailfish optimizer based Kapur's Thresholding (SFO-KT) technique is employed for image segmentation process. Also, feature extraction using Capsule Network (CapsNet) is derived to generate a set of feature vectors, and Political Optimizer (PO) with Cascade Forward Neural Network (CFNN) is applied to classify pancreatic tumors. A comprehensive experimental analysis is performed to highlight the improved outcome of the ODL-PTNTC technique and the results are inspected under several dimensions.

## 2. Related Works

This section provides a detailed review of existing pancreatic tumor classification models available in the literature. Ma et al. [10] focused on automatically identifying pancreas tumors in CT scans by creating a CNN classifier. A CNN method has been created by a dataset of 3494 CT scans attained from 3751 CT scans from 190 persons with normal pancreatic cancer and 222 persons with pathologically confirmed pancreas tumors. They determined 3 datasets from this image, estimated the method with respect to ternary classifiers (viz., tumor at head/neck of the pancreas, no tumor, and tumor at tail/body) and binary classifiers (viz., tumor or not) with tenfold cross validation, and evaluated the efficiency of the algorithm regarding the specificity, accuracy, and sensitivity.

In [11], a CNN-based DL method was employed for the CECT scans to attain three methods (arterial or venous, arterial, and venous methods), and the performance is estimated by an 8-fold cross validation method. The CECT image of the optimum stage is utilized to compare the TML and DL algorithms in forecasting the pathological grading of pNEN. The performances of radiotherapists with quantitative and qualitative CT results were also estimated. The optimal DL method from the 8-fold cross validation has been estimated on an independent testing set of nineteen people from Hospital II which is scanned on distinct scanners. Fu et al. [12] extended the RCF, presented to the fields of edge finding, for the difficult pancreatic segmentation and presented a new pancreatic segmentation network. Using multilayer upsampling architecture replacing the simplest upsampling operations in each stage, the presented network fully considered the multiscale comprehensive contexture data of objects (pancreas) to execute per-pixel segmentation. In addition, with the CT images, this network was trained and supplied, therefore attaining an efficient result.

Men et al. [13] proposed an end-to-end DDNN method for segmentation of this target. The presented method is an end-to-end architecture which enables faster testing and training. It contains 2 significant elements: a decoder network and an encoder network. The decoder network is employed for recovering the original resolution by positioning deconvolution and the encoder network is utilized for extracting the visual feature of healthcare images. An overall of 230 people identified with NPC stage I or II were added in this work. Xuan and You [9] introduced a DL-based HCNN for pancreas cancer diagnosis. An RNN was presented for meeting the problem of spatial discrepancy segmentation over slices of nearby images. The RNN produced CNN outcomes and fine-tuned the segmentation by improving the shape and smoothness. Further, the HCNN configuration and training objectives were demonstrated to the performances of pancreas cancer image segmentation.

Shen et al. [14] showed that a DL method trained for mapping prediction radiographs of a person to the respective three-dimensional anatomy could consequently generate volumetric tomographic X-ray images of the person from a single prediction view. They determined the possibility of the model with head-and-neck, upper-abdomen, and lung CT images from 3 people. Dmitriev et al. [15] determined an automated classification method which categorizes the 4 most popular kinds of pancreas cysts with CT scans. The presented method uses wide-ranging demographic data regarding the person and imaging presence of the cyst. It depends on a Bayesian integration of the RF classification that learns shape features, subclass specific demographics, and intensity, and a novel CNN method depends on fine texture data.

Manabe et al. [16] estimated an adapted CNN method for improving the performance of healthcare images. They adapted the CNN based AlexNet method using an input size of 512 × 512. They resized the filter size of max pooling and convolutional layers. With this adapted CNN, numerous methods were evaluated and created. The enhanced CNN was estimated for classifying the absence/presence of the pancreas in the CT scans. They related the total accuracy that is evaluated from images not utilized to train the ResNet. Boers et al. [8] performed the present interactive technique, iFCN, and proposed an interactive form of U-net technique called iUnet. iUnet is trained completely for producing the optimum initial segmentation. An interactive model is further trained on a partial set of layers on user-made scribbles. They compared primary segmentation performances of iUnet and iFCN on 100 CT datasets with dice similarity coefficient analysis.

## 3. The Proposed Model

In this study, an effective ODL-PTNTC technique is derived to detect and classify the existence of pancreatic tumors and nontumor. The proposed ODL-PTNTC technique encompasses different stages of operations such as AWF based preprocessing, SFO-KT based segmentation, CapsNet based feature extraction, CFNN based classification, and PO based parameter optimization. The design of SFO algorithm for optimal threshold value selection and PO based optimal selection of CFNN parameters results in enhanced classification performance.

### 3.1. AWF Based Preprocessing

Primarily, the AWF technique is utilized to remove the noise existing in the test images. To reduce the impulse noise, the standard MF could obtain a better outcome. But the standard MF has a fixed filter window; once a larger part of region gets affected by the impulse noise, it will be highly complex to obtain a better outcome. Further, once the amount of the noise pixels in the filter window is around half of the amount of each pixel, the MF algorithm will complete failure. For the above analysis, an adaptive filter window algorithm is adapted for filtering the impulse noise. As per the radio of pixels, they were impacted by the impulse noise in distinct areas, altering the filter window dimension. Assume that the first dimension of the filter window is *n* × *n* (*n* represents odd number), *m* represents amount of noise pixels in the window, and the extent was influenced by the impulse noise as

(1) $$\begin{array}{c} \gamma =\frac{m}{n\times n}\times 100\%. \end{array}$$

The adaptive MF is separated into parts a and b:

- The extent of effect: *γ* < T; then *S*_*i*,*j*_^*N*^=*S*_*i*,*j*_^*M*^=∑_*i*,*j*_^*S*^*S*/*τ*, *γ* ≥ *T*; jump to part b.
- Extent of the filter window: extend the filter window to $\left(\hat{n}+2\right)\times \left(\hat{n}+2\right)$, and reevaluate *γ*, and jump to part a.

Here, $\hat{n}\times \hat{n}$ represents the dimension of the latter filter window, *T* denotes the amount of the nonnoise pixel in the filter window, and *S*_*i*,*j*_^*M*^ indicates the median of nonnoise pixel in the filter window. *T* indicates the threshold of extent which was impacted by the impulse noise. In this case, the dimension of the MF window is fixed; once the quantity of the noise attains 3/10 of the number of the filter window pixels, the filter result changes to unacceptable. Hence, the *T* threshold is fixed at 0.3 for getting a better filter result [17]. The AWF algorithm advantage is given below:

- Since the AWF has the function to alter the dimension of the filter window based on the affected extent of the impulse noise, the complete failure of the MF is resolved, and the adaptive filter window is selected for getting a good filter outcome.
- The noise signal is filtered, and the effective signal that is not impacted by the impulse noise is maintained. During filtering, nonnoise pixels could perform the filter process, and the noise pixel is foreclosed. Next, it will reduce the effects of impulse noise on the filter outcome.
- Impulse noise pixel is filtered, and then, compared to standard MF, the speed is very high, and it will attain the feasibility of the method.

### 3.2. SFO-KT Based Segmentation Technique

During the image segmentation process, the SFO-KT technique receives the preprocessed image as input to determine the affected regions in the CT image. The idea of entropy criterion was presented by Kapur et al. in 1985 [18]. So far, it has been employed extensively in defining optimum threshold value in histogram‐based image segmentation. Like the Otsu model, initially, the entropy criterion was proposed for bilevel thresholding. It is expanded to resolve multilevel thresholding issues. It can be expressed by

(2) $$\begin{array}{c} H_{0}=-\overset{t}{\underset{i=0}{\sum }}\left(\frac{PR_{i}}{\omega_{0}}\right)ln\left(\frac{PR_{i}}{\omega_{0}}\right),H_{1}=-\overset{L-1}{\underset{i=t+1}{\sum }}\left(\frac{PR_{i}}{\omega_{1}}\right)ln\left(\frac{PR_{i}}{\omega_{1}}\right),\\ f_{Kapur}\left(t\right)=H_{0}+H_{1}, \end{array}$$

where *H*_0_ and *H*_1_ represent the entropy values of *C*_1_ and *C*_2_ and *f*_Kapur_(*t*) denotes the objective function. Assume a problem of defining *n* − 1 threshold; the multilevel thresholding can be expressed by

(3) $$\begin{array}{c} f_{Kapur}\left(t_{1}^{*},\;t_{2}^{*},\;\ldots ,\;t_{n-1}^{*}\right)=\max\left\{\overset{n-1}{\underset{i=1}{\sum }}H_{i}\right\}. \end{array}$$

This approach has been shown to be efficient for bilevel thresholding in image thresholding that is expanded to multilevel threshold for color and gray images. But the optimal threshold is derived by a thorough searching technique. It leads to a dramatic rise in the estimation time with the amount of thresholds. Therefore, assume the FF for gaining the optimum threshold {*t*_1_^*∗*^,  *t*_2_^*∗*^,   …,  *t*_*n*−1_^*∗*^} and an enhanced fruit fly optimization method is presented, which is employed to solve multilevel thresholding. A novel hybrid adoptive-cooperative learning approach is developed and a new solution system based on the idea that every dimension of the solution vector would be enhanced in one search to preserve the diverse population is presented. This method could efficiently reduce computational time, that is, mainly appropriate for multilevel image thresholding.

To optimally select the threshold values involved in Kapur's entropy, the SFO algorithm is utilized. The SFO is a new nature‐simulated metaheuristic technique that is inspired from the attack-alternation strategy of sailfish's group hunting [19]. It illustrates optimum efficiency related to popular metaheuristic approaches. During the SFO technique, sailfish can be regarded as candidate solution, the places of which under the exploration space signify the variable of issues. The place of *i*^th^ sailfish from the *k*^th^ search round was represented by *SF*_*i*,*k*_, and their equivalent fitness was evaluated by *f*(*SF*_*i*,*k*_). The sardines are another important participant under the SFO technique. It can be considered as school of sardines was also moving from the search spaces. The place of *i*^th^ sardine was demonstrated by *S*_*i*_, and its equivalent fitness was calculated by *f*(*S*_*i*_). During the SFO technique, the sailfish possessing the optimum place was chosen as elite sailfish that affects the manoeuvrability and acceleration of sardines under attack. Furthermore, the place of injured sardine under all the rounds is chosen as an optimum place for collaborative hunting by sailfish. This process aims at preventing previous discarding solution from being chosen again. Elite sailfish and injured sardines can be denoted as *Y*_new_*SF*__^*i*^, which refers the upgraded dependent upon the subsequent:

(4) $$\begin{array}{c} Y_{{\text{new}}_{SF}}^{i}=Y_{{\text{elite}}_{SF}}^{i}-\lambda_{i}\times \left(\text{random}\left(0,1\right)\times \left(\frac{Y_{{\text{elite}}_{SF}}^{i}-Y_{{\text{injured}}_{S}}^{i}}{2}\right)-Y_{{\text{current}}_{SF}}^{i}\right), \end{array}$$

where *Y*_currenT_*SF*__^*i*^ signifies the present place of sailfish and random (0,1) refers to the arbitrary number ranging between [0-1].

Variable *λ*_*i*_ defines the coefficient from the *i*^th^ iteration and its value is

(5) $$\begin{array}{c} \lambda_{i}=2\times \text{rand}\left(0,1\right)\times S\;D-S\;D, \end{array}$$

where *S*  *D* denotes the sardine density that signifies the amount of sardines under all the rounds. Variable *S*  *D* is resultant as

(6) $$\begin{array}{c} S\;D=1-\left(\frac{N_{SF}}{N_{SF}+N_{S}}\right), \end{array}$$

where *N*_*SF*_ and *N*_*S*_ stand for the amounts of sailfish and sardines correspondingly. Initially in the hunt, sailfish is energetic, and sardines are not tired/injured. The sardines escape quickly. But, with continuous hunting, the power of sailfish attack was slowly reduced. In the meantime, the sardines are developed tired, and their awareness of the place of sailfish is also reduced. Thus, the outcome is that the sardines are hunted. According to the algorithmic procedure, the new position of sardine *Y*_new_*S*__^*i*^ refers the upgraded dependent upon the subsequent:

(7) $$\begin{array}{c} Y_{new_{S}}^{i}=\text{random}\left(0,1\right)\times \left(Y_{elite_{SF}}^{i}-Y_{old_{S}}^{i}+ATP\right), \end{array}$$

where *Y*_old_*S*__^*i*^ signifies the old place of sardine and random (0,1) represents the arbitrary number ranging between [0-1]. *ATP* implies the sailfish attack power. Variable *ATP* was estimated as

(8) $$\begin{array}{c} ATP=B\times \left(1-\left(2\times ltr\times \varepsilon \right)\right), \end{array}$$

where *B* and *ε* stand for the coefficients utilized for reducing the attack power linearly in [*B*-0] and *Itr* represents the number of rounds. Since the attack power of sailfish reduces the hunting time, this reduction promotes the convergence of search. If *ATP* is higher, for instance, superior to 0.5, the place of all sardines is upgraded. Conversely, only *α* sardines with *β* variables upgrade their places. The number of sardines that upgrade their places is defined as

(9) $$\begin{array}{c} \alpha =N_{S}\times ATP, \end{array}$$

where *N*_*S*_ indicates the number of sardines under all the rounds. The number of variables of the sardines which upgrade their places is attained as

(10) $$\begin{array}{c} \beta =d_{i}\times ATP, \end{array}$$

where *d*_*i*_ represents the number of variables from the *i*^th^ round. If the sardine was hunted, its fitness could be superior to the sailfish. During this condition, the place of sailfish *Y*_*SF*_^*i*^ was upgraded with latest place of hunted sardine *Y*_*S*_^*i*^ for promoting the hunt for novel sardine. The equivalent formula is as follows:

(11) $$\begin{array}{c} Y_{SF}^{i}=Y_{S}^{i}\;if\;f\left(S_{i}\right)<f\left(SF_{i}\right). \end{array}$$

### 3.3. CapsNet Based Feature Extraction Technique

Once the images are segmented, the next stage is to derive a useful set of features using the CapsNet model. For resolving the limitations of CNN and generating it nearer to cerebral cortex activity framework, Hinton [20] presented a maximum dimension vector named “capsule” for representing an entity (object or part of object) with the set of neurons instead of single neuron. The performances of neurons within an active capsule signify different properties of specific entity that was projected from the image. All the capsules learned an understood explanation of visual entity which outcomes the probabilities of entity and the group of instantiated parameters including the precise pose (place, size, and orientation), hue, texture, deformation, albedo, and velocity.

The framework of CapsNet was distinct from those of other DL techniques. The outcomes of input as well as output of CapsNet were vectors if the norm and direction signify the existence probabilities and different attributes of entity correspondingly [21]. A similar level of capsule is utilized for predicting the instantiation parameter of superior level capsule with transformation matrix and, afterward, dynamic routing was implemented for making the forecast consistent. If the several forecasts are consistent, the superior level of one capsule is made active.  Figure 1 shows the structural overview of CapsNet model.

The framework was shallow through only 2 convolution layers (Convl, PrimaryCaps) and 1 fully connected (FC) layer (Entity‐Caps). In particular, Convl was a typical convolution layer that adapts images to main features and outputs to PrimaryCaps with convolutional filter through the size of 13 × 13 × 256. During the analysis, a novel image could not be appropriate to the input of primary layer of the CapsNet, as well as the rule features once convolution is implemented.

The secondary convolution layer makes the equal vector design as input of capsule layer. The typical convolutions of all outputs are scalar; however, the convolution of PrimaryCaps is distinct from the standard one. 2D convolution of 8 various weights to the input of 15 × 15 × 256 could be considered. Each time the implementation takes 32 sizes of 11 × 11 steps to 2 convolutions, and output 5 × 5 × 8 × 32 vector design input. The third layer (EntityCaps) was a resultant layer that involves 9 typical capsules equivalent to 9 various classes.

A layer of CapsNet was separated as to several calculation units called capsules. Let the capsule *i* output activities vector *u*_*i*_ in PrimaryCaps *i*; capsule *j* can be offered for generating activity level *v*_*j*_ of EntityCaps. Propagating and upgrading are conducted utilizing vectors among PrimaryCaps as well as EntityCaps. The matrix model was employed for scalar input from all the layers of typical NN that was importantly a linear group of outputs. The capsule model input was separated as to 2 steps, namely, linear combination and routing. The linear combination signifies the knowledge of modeling scalar inputs with NN that implies processing the connection among 2 objects from the scene with visual transformation matrix but preserving its concern. In detail, the linear combination is expressed as

(12) $$\begin{array}{c} {\hat{u}}_{ji}=u_{i}W_{ij}, \end{array}$$

where $\hat{u}$ signifies the forecast vector created by altering the outputs *u*_*i*_ of a capsule in the layer below by a weight *W*_*ij*_. Next, during the routing phase, the input vector *s*_*j*_ of capsule *j* is determined as

(13) $$\begin{array}{c} s_{j}=\sum_{i}c_{ij}{\hat{u}}_{j|i}, \end{array}$$

where *c*_*ij*_ refers to the coupling coefficient defined as iterative dynamic routing model. The routing part was really a weighted sum of $\hat{u}$ by the coupling coefficient. The vector outcome of capsule *j* was computed by implementing a nonlinear squashing function which is to make sure that short vector shrinks to nearly zero length and long vector obtained shrinks to length somewhat under one as

(14) $$\begin{array}{c} v_{j}=\frac{{\left\|s_{j}\right\|}^{2}}{1+{\left\|s_{j}\right\|}^{2}}\frac{s_{j}}{\left\|s_{j}\right\|}. \end{array}$$

Noticeably, the capsule activation function actually suppresses as well as redistributes vector lengths. The particular output was employed as probability of entities demonstrated as capsule from the present group. The entire loss function of novel CapsNet was a weighted summation of marginal loss and reconstruction loss. The MSE was utilized from the novel reconstruction loss function that degrades the model considerably if processing noisy data.

### 3.4. PO-CFNN Based Classification Model

During image classification process, the extracted features are fed into the CFNN model to allot proper class labels. The perceptron linking which is designed among input as well as output is created by direct connection but FFNN links generated among input as well as output are by indirect connection. The connection was nonlinear from shape with activation function under the hidden layer. When the association procedure on perceptron and multilayer network are joined, the input and output layers are linked in an indirect way [22]. The network made in this connection design is named CFNN. The formula generated in CFNN technique is expressed as

(15) $$\begin{array}{c} y=\overset{n}{\underset{i=1}{\sum }}f^{i}\omega_{i}^{i}x_{i}+f^{o}\left(\overset{k}{\underset{j=1}{\sum }}\omega_{j}^{o}f_{j}^{h}\left(\overset{n}{\underset{i=1}{\sum }}\omega_{ji}^{h}x_{i}\right)\right), \end{array}$$

where *f* stands for the activation function under the input-output layers and *ω*_*i*_^*i*^ implies the weight in the input-output layers. When the bias was more to input layer and activation function of all neurons under the hidden layer is *f*^*h*^,

(16) $$\begin{array}{c} y=\overset{n}{\underset{i=1}{\sum }}f^{i}\omega_{i}^{i}x_{i}+f^{o}\left(\omega^{b}+\overset{k}{\underset{j=1}{\sum }}\omega_{j}^{o}f^{h}\left(\omega_{j}^{b}+\overset{n}{\underset{i=1}{\sum }}\omega_{ji}^{h}x_{i}\right)\right). \end{array}$$

During this investigation, the CFNN technique was executed from time series data. So, the neuron from the input layer is delayed time series data *X*_*t*−1_, *X*_*t*−2_,…, *X*_*t*−*p*_, while the output was present data *X*_*t*_. The overall structure of CFNN model is shown in Figure 2.

For optimally selecting the parameters involved in the CFNN model, the PO algorithm is applied to it. PO algorithm is a current metaheuristic method proposed by Askari et al. It is stimulated by the political method with multiphase nature [23]. Politics is based on the political struggles among 2 individuals; every individual tries to improve their goodwill to win the election. All the parties try to expand the number of seats in parliament to the maximal range to form the government. In PO, the member of the parties is assumed as an individual (candidate solution) when the individual goodwill is assumed as the candidate solution location (design variable). The election signifies the objective function, that is, determined according to the number of votes attained by the candidate. The party formation, PO, electioneering, parliamentary affairs, distribution of constituencies, elections within the party, and party switching are the seven stages of the parliament. The initial stage can be executed one time; it is assumed as initiation procedure when the other stages are executed in loop.  Figure 3 shows the flowchart of PO algorithm.

In the party distribution stage, the population comprises *n* parties, all the parties have *n* members (candidates), and all the candidates are denoted as a *d*‐dimension vector. It can be expressed mathematically by

(17) $$\begin{array}{c} P=\left\{P_{1},P_{2},P_{3},\;\ldots ,P_{n}\right\},\\ P_{i}=\left\{p_{i}^{1},p_{i}^{2},p_{i}^{3},\ldots ,p_{i}^{n}\right\},\\ p_{i}^{j}={\left[p_{i,1}^{j},p_{i,2}^{j},p_{i,3}^{j},\ldots ,p_{n}^{j}\right]}^{T}. \end{array}$$

In the above formula, *Pn* represents the *n*th political party and *p*_*i*_^*n*^ denotes the *n*th candidate member. In addition, there are *n* precincts; all the party members contest the election from the precincts as follows:

(18) $$\begin{array}{c} c=\left\{c_{1},\;c_{2},\;c_{3},\;c_{n}\right\},\\ c_{j}=\left\{p_{1}^{j},p_{2}^{j},p_{3}^{j},\ldots ,p_{n}^{j}\right\}. \end{array}$$

The fittest party members are assumed as the leader; this can be announced after the election inside the party as

(19) $$\begin{array}{c} q=\text{ arg min}f\left(p_{i}^{j}\right),\;\forall i\in \left\{1,2,\;\ldots .n\right\},\\ p_{i}^{*}=p_{i}^{q}. \end{array}$$

Let *p*_*i*_^*∗*^ be the *i*th party leader and *f*(*p*_*i*_^*j*^) represents the fitness function of *p*_*i*_^*j*^. The vectors signifying each leader are formulated by

(20) $$\begin{array}{c} P^{*}=\left\{p_{1}^{*},p_{2}^{*},p_{3}^{*},\;\ldots ,p_{n}^{*}\right\}. \end{array}$$

The vector of each parliamentarian is expressed by

(21) $$\begin{array}{c} c^{*}=\left\{c_{1}^{*},\;c_{2}^{*},\;c_{3}^{*},\;c_{n}^{*}\right\}, \end{array}$$

where *c*_*j*_^*∗*^ represents the *j*th constituency winner. The electioneering phase allows the candidate to improve their performances in the electoral procedure; it can be performed by 3 characteristics: comparative analysis with the winner, learning from the prior election, and effects of vote bank that the party leader gained. The initial one is modeled by an approach of upgrading previous location as

(22) $$\begin{array}{c} p_{i,k}^{j}\left(t+1\right)=\left\{\begin{array}{cc} m^{*}+r\left(m^{*}-p_{i,k}^{j}\left(t\right)\right)\;, & p_{i,k}^{j}\left(t-1\right)\leq {\text{p}}_{i,k\;}^{\text{j}}\left(t\right)\leq m^{*}or{\text{ p}}_{i,k}^{\text{j}}\left(t-1\right)\geq p_{i,k}^{j}\left(t\right)\geq m^{*},\\ m^{*}+\left(2r-1\right)\left|m^{*}-{\text{p}}_{i,k}^{\text{j}}\left(t\right)\right|, & {\text{p}}_{i,k}^{\text{j}}\left(t-1\right)\leq m^{*}\leq p_{i,k}^{j}\left(t\right)\;or\;p_{i,k}^{j}\;\left(t-1\right)\geq m^{*}\geq p_{i,k}^{j}\left(t\right),\\ m^{*}+\left(2r-1\right)\left|m^{*}-p_{i,k}^{j}\left(t-1\right)\right| & m^{*}\leq p_{i,k}^{j}\left(t-1\right)\leq p_{i,k}^{j}\left(t\right)\;or\;m^{*}\geq p_{i,k}^{j}\left(t-1\right)\geq p_{i,k}^{j}\left(t\right), \end{array}\right.\\ p_{i,k}^{j}\left(t+1\right)=\left\{\begin{array}{cc} m^{*}+\left(2r-1\right)\left|m^{*}-p_{i,k}^{j}\left(t\right)\right|, & p_{i,k}^{j}\left(t-1\right)\leq {\text{p}}_{i,k\;}^{\text{j}}\left(t\right)\leq m^{*}or{\text{ p}}_{i,k}^{\text{j}}\left(t-1\right)\geq p_{i,k}^{j}\left(t\right)\geq m^{*},\\ p_{i,k}^{j}\left(t-1\right)+r\left(p_{i,k}^{j}\left(t\right)-{\text{p}}_{i,k}^{\text{j}}\left(t-1\right)\right), & {\text{p}}_{i,k}^{\text{j}}\left(t-1\right)\leq m^{*}\leq p_{i,k}^{j}\left(t\right)\;or\;p_{i,k}^{j}\;\left(t-1\right)\geq m^{*}\geq p_{i,k}^{j}\left(t\right),\\ m^{*}+\left(2r-1\right)\left|m^{*}-p_{i,k}^{j}\left(t-1\right)\right| & m^{*}\leq p_{i,k}^{j}\left(t-1\right)\leq p_{i,k}^{j}\left(t\right)\;or\;m^{*}\geq p_{i,k}^{j}\left(t-1\right)\geq p_{i,k}^{j}\left(t\right), \end{array}\right. \end{array}$$

where *r* represents an arbitrary number within [0,1]; *p*_*i*,*k*_^*j*^(*t*) signifies the location of *j*th candidate of *j*th political party at *t* iteration, and *m*^*∗*^ is k‐dimension vector holding *p*_*i*_^*∗*^ and dealing with *c*_*j*_^*∗*^. The above equations are applied for updating the candidate location according to the relationships among the present FF and the prior one. Meanwhile the FF is enhanced when it is located once the fitness is degraded.

The party switching stage can be performed by allocating a variable called party switch rate (*λ*); it is initiated by *λ*_max_ and linearly reduced to 0 at the time of iteration process. All the members have a likelihood value of *λ* according to the switching to (*p*_*r*_^*j*^) random party which is carried out, and the member could be exchanged by the worst fit member (*p*_*r*_^*q*^). The *q* index is estimated by

(23) $$\begin{array}{c} q=\text{argmax }f\left(p_{r}^{j}\right),\\ 1\leq j\leq n. \end{array}$$

The election is imitated by measuring the fitness of each individual competing candidate in the electoral district and announcing the winner according to the succeeding equation:

(24) $$\begin{array}{c} q=\text{arg}\;\text{min }f\left({\text{p}}_{i}^{\text{j}}\right),\forall i\in \left\{1,2,\;\ldots .n\right\}\\ c_{j}^{*}=p^{j_{q}}, \end{array}$$

where *c*_*j*_^*∗*^ represents the *jth* constituency winner, and the leader of the party is upgraded by equation (24).

After implementing the election inside the party, the government is created. The parliamentarian is explained by equations (18) and (23). In this stage, the parliamentarians update their location, while the assessed FF values are optimized.

## 4. Experimental Validation

In this section, the pancreatic tumor classification performance of the ODL-PTNTC technique is investigated using the benchmark BioGPS dataset from [9]. The dataset comprises CT images and a sample set of images are shown in Figure 4. The results are inspected under different training sizes (TS) and folds (*K*).

Table 1 and Figure 5 offer a detailed comparative classification results analysis of the ODL-PTNTC technique with existing techniques under diverse TS. With TS = 40%, the proposed ODL-PTNTC technique has attained a higher sens_*y*_ of 99.89%, whereas the DS-WELM, DS-KELM, and DS-ELM techniques have obtained lower sens_*y*_ of 99.69%, 96.97%, and 96.79%, respectively. In addition, with TS = 40%, the projected ODL-PTNTC manner has gained a superior spec_*y*_ of 96.96%, whereas the DS-WELM, DS-KELM, and DS-ELM methodologies have obtained lower spec_*y*_ of 96.22%, 96.87%, and 96.96% correspondingly. At the same time, with TS = 40%, the proposed ODL-PTNTC manner has achieved a superior accu_*y*_ of 96.96%, whereas the DS-WELM, DS-KELM, and DS-ELM methods have obtained decreased accu_*y*_ of 96.22%, 96.87%, and 96.96% correspondingly. Likewise, with TS = 40%, the presented ODL-PTNTC system has attained an enhanced *F*_score_ of 98.92%, whereas the DS-WELM, DS-KELM, and DS-ELM algorithms have obtained minimum *F*_score_ of 98.39%, 98.59%, and 94.32% correspondingly.

Table 2 and Figure 6 report the overall average classification results analysis of the ODL-PTNTC technique. The results demonstrated that the ODL-PTNTC technique has resulted in maximum classification performance under distinct TS. The obtained values highlighted that the ODL-PTNTC technique has gained improved outcomes with sens_*y*_, spec_*y*_, accu_*y*_, and *F*_score_ of 98.73%, 97.75%, 98.40%, and 98.82%, respectively.

Table 3 and Figure 7 provide a detailed comparative classification outcomes analysis of the ODL-PTNTC system with existing algorithms under diverse *K* folds. With *K* = 6, the presented ODL-PTNTC method has attained maximal sens_*y*_ of 97.73%, whereas the DS-WELM, DS-KELM, and DS-ELM systems have obtained lower sens_*y*_ of 97.57%, 96.07%, and 94.31% correspondingly. Likewise, with *K* = 6, the proposed ODL-PTNTC scheme has attained maximum spec_*y*_ of 99.42% but the DS-WELM, DS-KELM, and DS-ELM techniques have obtained lower spec_*y*_ of 99.27%, 96.25%, and 98.03% correspondingly. With *K* = 6, the projected ODL-PTNTC technique has reached increased accu_*y*_ of 99.77%, whereas the DS-WELM, DS-KELM, and DS-ELM manners have obtained lower accu_*y*_ of 98.46%, 99.34%, and 93.79%, respectively. In addition, with *K* = 6, the presented ODL-PTNTC technique has obtained superior *F*_score_ of 98.24%, whereas the DS-WELM, DS-KELM, and DS-ELM methodologies have reached decreased *F*_score_ of 97.99%, 98.1%, and 96.57% correspondingly.

Table 4 and Figure 8 illustrate the overall average classification outcomes analysis of the ODL-PTNTC manner. The outcomes indicate that the ODL-PTNTC manner has resulted in maximal classification performance in several *K* folds. The reached values exhibited that the ODL-PTNTC methodology has attained increased outcome with sens_*y*_,  spec_*y*_, accu_*y*_, and *F*_score_  of 97.88%, 99.38%, 98.08%, and 98.63%, respectively.

A wide-ranging comparative classification results analysis of the ODL-PTNTC technique with recent approaches is given in Table 5 [24, 25].

Figure 9 examines the relative sens_*y*_  analysis of the ODL-PTNTC approach with existing manners. The outcomes demonstrated that the CNN-10 × 10, CNN-30 × 30, CNN-50 × 50, CNN-70 × 70, and EEDL-DPT methods have reached minimal sens_*y*_ values of 80.50%, 88.10%, 91.10%, 91.50%, and 61.95% correspondingly. Simultaneously, the DS-ELM, DS-KELM, DL-HCNN, and CNN-CTPCD systems have obtained moderate sens_*y*_ values of 96.27%, 96.66%, 97.66%, and 91.58% correspondingly. However, the DS-WELM algorithm has accomplished near optimal sens_*y*_  of 97.76%, and the projected ODL-PTNTC method has resulted in maximal sens_*y*_ of 98.73%.

Figure 10 explores the comparative spec_*y*_  analysis of the ODL-PTNTC approach with recent techniques. The outcomes demonstrated that the CNN-10 × 10, CNN-30 × 30, CNN-50 × 50, CNN-70 × 70, and EEDL-DPT methods have reached lesser spec_*y*_ values of 81.80%, 85.40%, 86.50%, 86.50%, and 90.20% correspondingly. Besides, the DS-ELM, DS-KELM, DL-HCNN, and CNN-CTPCD techniques have attained moderate spec_*y*_ values of 97.27%, 97.53%, 96.12%, and 98.27% correspondingly. Also, the DS-WELM manner has accomplished near optimal spec_*y*_  of 97.75%, and the presented ODL-PTNTC technique has resulted in increased spec_*y*_ of 97.75%.

Figure 11 investigates the comparative accu_*y*_ analysis of the ODL-PTNTC technique with recent approaches. The results depicted that the CNN-10 × 10, CNN-30 × 30, CNN-50 × 50, CNN-70 × 70, and EEDL-DPT techniques have obtained lower accu_*y*_ values of 81.60%, 85.90%, 87.30%, 87.040%, and 82.70%, respectively. At the same time, the DS-KELM, DS-ELM, DL-HCNN, and CNN-CTPCD techniques have attained moderate accu_*y*_ values of 96.69%, 96.21%, 96.89%, and 95.47%, respectively. Though the DS-WELM technique has accomplished near optimal accu_*y*_  of 97.26%, the proposed ODL-PTNTC technique has resulted in maximum accu_*y*_ of 98.40%.

Finally, an ROC analysis of the ODL-PTNTC technique on the test dataset is shown in Figure 12. The results demonstrated that the ODL-PTNTC technique has resulted in maximum ROC of 99.6723. From the above results and discussion, it is evident that the ODL-PTNTC technique has accomplished improved pancreatic tumor classification performance.

## 5. Conclusion

In this study, an effective ODL-PTNTC technique is derived to detect and classify the existence of pancreatic tumors and nontumor. The proposed ODL-PTNTC technique encompasses different stages of operations such as AWF based preprocessing, SFO-KT based segmentation, CapsNet based feature extraction, CFNN based classification, and PO based parameter optimization. The design of SFO algorithm for optimal threshold value selection and PO based optimal selection of CFNN parameters results in enhanced classification performance. For examining the improved outcomes of the ODL-PTNTC technique, a series of simulations take place and the results are investigated under numerous aspects. A wide-ranging comparative results analysis stated the superior efficiency of the ODL-PTNTC technique compared to the recent approaches. In the future, the DL based segmentation techniques can be designed to improve the classification performance of the ODL-PTNTC technique.

## Figures and Tables

**Figure 1:** Structure of CapsNet model.

**Figure 2:** Overview of CFNN model.

**Figure 3:** Flowchart of PO algorithm.

**Figure 4:** Sample images.

**Figure 5:** Result analysis of ODL-PTNTC model under different TS.

**Figure 6:** Overall result analysis of ODL-PTNTC model under different TS.

**Figure 7:** Result analysis of ODL-PTNTC model under different *K* folds.

**Figure 8:** Overall result analysis of ODL-PTNTC model under different *K* folds.

**Figure 9:** Sensitivity analysis of ODL-PTNTC technique with existing manners.

**Figure 10:** Specificity analysis of ODL-PTNTC technique with existing manners.

**Figure 11:** Accuracy analysis of ODL-PTNTC technique with existing manners.

**Figure 12:** ROC analysis of ODL-PTNTC technique.

**Table 1:** Comparative classification results analysis of ODL-PTNTC technique under varying training set (TS).

Training (%)	ODL-PTNTC	DS-WELM	DS-KELM	DS-ELM
*Sensitivity*				
TS = 40	99.89	99.69	96.97	96.79
TS = 50	98.55	98.35	98.23	97.49
TS = 60	98.32	97.20	98.00	97.12
TS = 70	97.59	96.53	97.02	97.13
TS = 80	99.31	98.89	97.82	96.28
**Average**	**98.73**	**98.13**	**97.61**	**96.96**

*Specificity*				
TS = 40	96.96	96.22	96.87	96.96
TS = 50	97.20	96.84	97.12	95.43
TS = 60	98.82	98.70	95.78	97.78
TS = 70	97.57	96.46	97.19	95.31
TS = 80	98.18	97.53	97.64	97.74
**Average**	**97.75**	**97.15**	**96.92**	**96.64**

*Accuracy*				
TS = 40	98.34	98.29	95.44	97.46
TS = 50	99.08	97.60	97.92	98.93
TS = 60	98.50	98.47	94.87	94.59
TS = 70	97.21	96.52	97.02	94.32
TS = 80	98.86	97.42	98.37	96.90
**Average**	**98.40**	**97.66**	**96.72**	**96.44**

*F-score*				
TS = 40	98.92	98.39	98.59	94.32
TS = 50	99.08	95.76	98.84	96.51
TS = 60	99.84	99.70	97.10	97.08
TS = 70	98.27	96.71	95.55	97.88
TS = 80	97.98	96.40	94.31	97.93
**Average**	**98.82**	**97.39**	**96.88**	**96.74**

**Table 2:** Overall classification results analysis of ODL-PTNTC technique under varying training size (TS).

Measures	Methods			
	ODL-PTNTC	DS-WELM	DS-KELM	DS-ELM
Sensitivity	98.73	98.13	97.61	96.96
Specificity	97.75	97.15	96.92	96.64
Accuracy	98.40	97.66	96.72	96.44
*F*-score	98.82	97.39	96.88	96.74

**Table 3:** Comparative classification results analysis of ODL-PTNTC technique under varying *K* folds.

No. of folds	ODL-PTNTC	DS-WELM	DS-KELM	DS-ELM
*Sensitivity*				
*K* = 6	97.73	97.57	96.07	94.31
*K* = 7	97.61	96.03	96.54	97.41
*K* = 8	98.53	98.29	94.45	97.48
*K* = 9	96.70	96.44	96.05	93.75
*K* = 10	98.85	98.59	95.46	94.89
**Average**	**97.88**	**97.38**	**95.71**	**95.57**

*Specificity*				
*K* = 6	99.42	99.27	96.25	98.03
*K* = 7	98.80	98.57	96.72	98.51
*K* = 8	99.45	96.99	98.72	99.37
*K* = 9	99.75	98.22	99.65	96.50
*K* = 10	99.47	97.88	99.32	97.06
**Average**	**99.38**	**98.19**	**98.13**	**97.89**

*Accuracy*				
*K* = 6	99.77	98.46	99.34	93.79
*K* = 7	99.44	96.98	99.04	97.46
*K* = 8	96.23	95.46	96.10	94.22
*K* = 9	96.48	96.18	94.86	96.09
*K* = 10	98.47	97.15	93.89	98.29
**Average**	**98.08**	**96.85**	**96.65**	**95.97**

*F-score*				
*K* = 6	98.24	97.99	98.1	96.57
*K* = 7	98.32	97.96	97.44	96.15
*K* = 8	98.05	97.84	97.64	96.92
*K* = 9	99.92	95.78	97.86	99.87
*K* = 10	98.63	98.21	95.31	96.00
**Average**	**98.63**	**97.56**	**97.27**	**97.10**

**Table 4:** Overall classification results analysis of ODL-PTNTC technique under varying *K* folds.

Measures	Methods			
	ODL-PTNTC	DS-WELM	DS-KELM	DS-ELM
Sensitivity	97.88	97.38	95.71	95.57
Specificity	99.38	98.19	98.13	97.89
Accuracy	98.08	96.85	96.65	95.97
*F*-score	98.63	97.56	97.27	97.10

**Table 5:** Comparative analysis of ODL-PTNTC technique with existing approaches.

Methods	Sensitivity	Specificity	Accuracy
ODL-PTNTC	98.73	97.75	98.40
DS-WELM	97.76	97.67	97.26
DS-KELM	96.66	97.53	96.69
DS-ELM	96.27	97.27	96.21
CNN-10 × 10	80.50	81.80	81.60
CNN-30 × 30	88.10	85.40	85.90
CNN-50 × 50	91.10	86.50	87.30
CNN-70 × 70	91.50	86.70	87.40
EEDL-DPT	61.95	90.20	82.70
DL-HCNN	97.66	96.12	96.89
CNN-CTPCD	91.58	98.27	95.47

## Data Availability

Data sharing is not applicable to this article as no datasets were generated during the current study.
